# Political uses of the ancient past on social media are predominantly negative and extreme

**DOI:** 10.1371/journal.pone.0308919

**Published:** 2024-09-04

**Authors:** Chiara Bonacchi, Jessica Witte, Mark Altaweel

**Affiliations:** 1 Department of Archaeology, School of History, Classics and Archaeology, University of Edinburgh, Edinburgh, United Kingdom; 2 Institute of Archaeology, University College London, London, United Kingdom; CCET: Chandigarh College of Engineering and Technology, INDIA

## Abstract

This study assesses whether references to the ancient past in debates about political issues on social media over-represent negative and extreme views. Using precision-recall, we test the performance of three sentiment analysis methods (VADER, TextBlob and Flair Sentiment) on a corpus of 1,478,483 posts, comments and replies published on Brexit-themed Facebook pages between 2015 and 2017. Drawing on the results of VADER and manual coding, we demonstrate that: 1) texts not containing keywords relating to the Iron Age, Roman and medieval (IARM) past are mostly neutral and 2) texts with IARM keywords express more negative and extreme sentiment than those without keywords. Our findings show that mentions of the ancient past in political discourse on multi-sided issues on social media are likely to indicate the presence of hostile and polarised opinions.

## 1. Introduction

For centuries, the past has been leveraged as a powerful means of framing and legitimising political identities [1–4]. Today, such identities are often expressed on social media. However, most of the existing literature on political uses of the past online has analysed populist nationalist and Far-Right speech [5–9]. Very few studies have examined how references to the past feature in multi-sided discussions about a specific political issue [10, 11]. Therefore, although substantial knowledge outlines how different ‘myths’ and heritage symbols are invoked to support extreme ideologies in online environments, there is virtually no information on whether people with more moderate views similarly mobilise the past to make sense of the present and plan for the future. The philosopher Jon Rüsen defines historical consciousness as the ‘mental procedure by which the past is interpreted for the sake of understanding the present and anticipating the future’ [12 p. 45]. Studying historical consciousness not only in the context of nationalism and extremism, but also in social media debates about political issues between users with more nuanced or milder opinions, is key to fully grasping how conceptions of the past shape political identities and decision-making.

Furthermore, researchers have yet to formally investigate the significance of sentiment polarity and its extremity, or strength of polarity, in relation to social media users’ positions in heritage-based political debates. Some research has speculatively reflected on the relationship between emotions, historical thinking and political activism online [8, 11]. This scholarship highlighted several *topoi* present in populist and far-right discourse referencing the past on Twitter/X: threat to the ingroup and their heritage; a quest for justice for those who belong to the ingroup; and heroism and collective action to restore justice for the ingroup [7, 11, 13, 14]. This literature also specifically stressed that heritage on social media is used to create affective ingroups ‘along religious-cultural lines’ that exclude those who do not belong [8, 14]. However, existing studies do not rigorously measure the polarity and extremity of this ‘affective’ dimension. Yet detecting negatively polarised sentiment can be useful for identifying and combatting hostility linked with extremism and ‘group-based anger’ online [15].

Extremist speech can be hidden using seemingly neutral language [16]. More frequently, however, extremity in ideology is positively correlated with extremity in sentiment polarity. As Weismueller and colleagues have shown, Twitter/X users with politically extreme views tend to share strongly negative content more frequently than those who hold moderate opinions [17]. In turn, tweets displaying extreme sentiment correlate with a higher number of retweets [17], especially if they have negative polarity [18]. Furthermore, some research suggests that communities on social media function as negatively polarised ‘echo chambers’ where users holding similar opinions discuss topics amongst each other, rarely encountering different beliefs. For example, in examining the consumption of Brexit-related information on news media Facebook pages, Del Vicario et al. found ‘two distinct communities of news outlets’ where individuals did not interact with the opposing viewpoint and expressed content with primarily negative sentiment [19 p. 6]. However, other research has concluded that the “echo chamber” effect might be overstated. For instance, participants in multi-sided discussion online still develop polarised perspectives as a result of exchanging emotionally heightened content [20]. Texts of this kind trigger motivated reasoning, a bias ‘directly related to ideological beliefs’ such as those ‘which signify and promote loyalty to an in-group’ [21 p. 5]. In turn, motivated reasoning leads to opinion polarisation [20].

Our study examines whether the Iron Age, Roman and early medieval (IARM) past is leveraged to express overtly negative and extreme political views. We address these questions through conducting a sentiment analysis on a corpus of posts, comments and replies collected from public Facebook pages related to the 2016 Referendum on the UK’s membership of the European Union. The absence of comparable formal assessments of sentiment in heritage studies does not allow us to formulate clear hypotheses. Furthermore, the more speculative literature available on the affective power of heritage in political discourse online focuses on Far Right and extreme nationalist ideologies. Given the impossibility of making directional predictions, we will explore whether texts referencing the IARM past in multi-sided social media discussions about Brexit will be:

1. prevalently negative and extreme;
2. more negative and extreme than content not containing mentions of the ancient past.

## 2. Materials and methods

### 2.1. Materials

The dataset consists of a corpus of 1,478,483 posts, comments and replies published in English on 364 public Facebook pages that had the word ‘Brexit’ in the title or description. These documents were extracted from 1 March to 30 April 2017 using Facebook’s public API; they were anonymised by substituting usernames and IDs with random numbers. Within the corpus, we identified a subset of 2,528 documents containing at least one reference to the Iron Age, Roman and early medieval (IARM) past of Britain via a keyword-based approach. IARM heritage keywords comprised place names, names of key historical figures and terms used to refer to the period between 800 BCE and 800 CE. The detection of keywords was undertaken as part of prior research (for details on how it was conducted, see [22, p. 178]). We chose the Natural Language Toolkit (NLTK) library in Python to prepare the corpus for sentiment analysis by performing word tokenisation and removing English-language stop words, non-ASCII characters (e.g. punctuation and symbols such as &, %,?) and extra white spaces.

This corpus comprises Facebook pages and, within them, views representing different positions towards Brexit, with some being in favour and others against [10]. It was compiled as part of previous research [10, 11], but ethical approval for new analyses was sought and obtained in 2022 from the University of Edinburgh. We chose to analyse our existing dataset for two reasons. First, examining social media data about Brexit, a high-profile event that has been intensely studied, offers significant opportunities for comparing our findings to existing work whilst contributing to ongoing scholarship on public discourse about political phenomena. Second, in the UK and in many other countries, institutional ethics policies require researchers to acquire data in compliance with platforms’ Terms of Service (ToS) agreements. Like other major platforms including X (formerly Twitter), Instagram and TikTok, Facebook’s ToS state that data must be extracted using its application programming interface (API). Yet following the Cambridge Analytica scandal, Facebook closed its public API, making it challenging to acquire additional data from the platform. Although the so-called ‘post-API age’ may appear to introduce a new barrier to reproducibility in studies examining social media data, such research has always been difficult to reproduce due to a host of known quality issues from platform-sourced data. However, despite these limitations, it is critical to continue studying social media data in acknowledgment that platforms function as public spaces for discourse on a range of political topics.

### 2.2. Background to methods

Sentiment analysis is a natural language processing (NLP) approach for studying human emotion in text [23]. Recently created frameworks allow measurements of both sentiment polarity, that is a negative, positive, or neutral orientation, and extremity, which is defined as overall strength of sentiment. Such frameworks have been used to examine a variety of textual data [24, 25]. Sentiment analysis methods can be subdivided into three distinct groups. The first consists of dictionary-based methods, which pair keywords (or phrases) with corresponding emotion or polarity values [26, 27]. For example, Almatarneh and Gamallo applied a lexicon-based method to assess extreme opinions, defined as the most positive or negative [26]. Similarly, Heidenreich and colleagues utilised a dictionary to examine the level of extreme sentiment in status updates about migration published by the Facebook accounts of 1702 political actors [27].

The second group of frameworks relies on machine learning. In this case, sentiment is investigated with the support of vector machines (SVM), Naive Bayes (NB), deep learning techniques including artificial neural networks, and regression-based methods [28, 29]. For instance, Sofat and Bansal chose multiple methods, including convolutional neural network long short-term memory (CNN-LSTM), to detect radical content in tweets and blog posts [30]. Jamil and co-authors identified extreme sentiment with the language representation model BERT (Bidirectional Encoder Representations from Transformers), which facilitates context awareness in determining word meanings, thereby improving score accuracy [31].

Finally, a third approach to sentiment analysis combines dictionary-based and machine learning methods [32–34]. The results of individual methods are deemed stronger if other techniques lead to comparable conclusions or one method can be shown to support higher accuracy and consistency for desired predictions. Dictionaries are flexible and adaptable, providing the possibility to analyse specific thematic domains with bespoke sets of keywords. On the other hand, machine learning techniques report relatively higher accuracy and precision, but require the creation of a sufficiently large training corpus [35–37].

### 2.3. Methods

As prior work has highlighted, a multi-method approach to identifying sentiment most accurately captures both polarity and extremity relative to the subject and linguistic features of the corpus. Therefore, we initially chose this strategy, deploying and subsequently testing the accuracy of VADER (Valence Aware Dictionary for sEntiment Reasoning), TextBlob Sentiment, and Flair Sentiment. We selected these specific techniques because they have an established track record of being deployed in comparable studies, which we discuss below. The code used to undertake the analysis is available via GitHub [38].

Both VADER and TextBlob are dictionary-based methods. VADER maps lexical features to emotional intensities providing sentiment scores from -1 (negative) to 1 (positive), with 0 being neutral [39–42]. TextBlob also incorporates aspect-based sentiment analysis, that is tools to identify the subject target and sentiment polarity [41]. This was evaluated in our initial search for methods to compare along with the other libraries of TextBlob. For our results, aspect-based sentiment was not seen as the key focus as we attempted to capture more general sentiment. Finally, Flair Sentiment [43, 44] uses an LSTM neural network model and multiple embedding types (GloVe, BERT, and ELMo) to contextualise the sentiment of terms based on their surrounding text. Sentences are scored between 0 and 1, with ‘negative’ or ‘positive’ designations. It is possible to train the LSTM neural network with either a bespoke corpus created by the user or a standard pre-trained library. We tried both approaches and, surprisingly, found the latter to be more accurate and sensitive than training with a bespoke corpus. This was likely due to the size of the subset of our corpus containing IARM keywords, which was too small for satisfactory training.

To establish which sentiment analysis technique might generate results consistent with empirical evidence, we compared the outputs of the different analyses discussed above using 500 randomly sampled texts without keywords (Sample 1) and 300 with keywords (Sample 2). Neither sample included neutrally polarised texts. Sample 2 comprised 300 texts because these were the ones available for coding once neutrals had been excluded (Sample 2). Thereafter, we performed precision and recall tests on these samples to obtain accuracy measures for positive predictions and sensitivity, or completeness [45]. Precision, recall and F1 scores were initially calculated for positive and negative sentiment and, subsequently, for extreme (>0.75 or <-0.75) and mild sentiment (<0.75 or >-0.75). The results of this analysis were split into categories based on validity and polarity: true extreme positive, false extreme positive, true mild positive, false mild positive, true extreme negative, false extreme negative, true mild negative and false mild negative.

## 3. Results

In this section, we present the results of the precision and recall tests on randomised values. We then discuss the polarity scores of the most accurate method when applied to the corpus of Brexit-themed public Facebook pages. Finally, we integrate this analysis with the outcomes of manual coding of randomly selected documents from Sample 1 (without IARM heritage keywords) and Sample 2 (with IARM heritage keywords).

### 3.1 Precision-recall results

Overall, the precision and recall tests demonstrate that the different approaches to sentiment analysis can reliably detect general negative or positive sentiment in texts that do not contain mentions of the IARM past (Sample 1), but are less successful in capturing sentiment extremity (Table 1). Additionally, we find that precision and recall for texts with IARM heritage keywords (Sample 2) is much weaker. For Sample 1, VADER and Lexical term lists scored highest in the Positive-Negative precision and recall tests, while VADER and Flair scored highest for Extreme-Non-Extreme tests. Therefore, when considering the results of all tests together, VADER is the most accurate and the most sensitive for analysing texts with no mentions of the IARM past.

**Table 1:** Precision-recall tests for negative and positive sentiment, and for extreme and non-extreme sentiment, applied to Sample 1 and Sample 2.

Test	Precision-Recall	Flair	VADER	TextBlob	Lexical
Positive-Negative (Sample 1)	Precision	0.57	0.81	0.74	0.79
	Recall	0.71	0.86	0.81	0.94
	F1 Score	0.63	0.83	0.78	0.86
Extreme and Non-Extreme (Sample 1)	Precision	0.47	0.55	0.37	0.32
	Recall	0.65	0.71	0.54	0.54
	F1 Score	0.54	0.62	0.44	0.4
Positive-Negative (Sample 2)	Precision	0.23	0.13	0.14	0.08
	Recall	0.19	0.11	0.20	0.15
	F1 Score	0.21	0.12	0.16	0.11
Extreme and Non-Extreme (Sample 2)	Precision	0.23	0.25	0.47	0.22
	Recall	0.19	0.22	0.44	0.26
	F1 Score	0.21	0.23	0.45	0.23

### 3.2 VADER results

Because VADER displayed the best overall precision-recall scores for Sample 1, we utilised the method for the full analysis of 974,053 posts, comments and replies that do not reference the IARM past. The precision-recall suggests a lower precision for extremity measures than polarity measures in all methods, including VADER. Therefore, we will discuss the total counts for negative, positive, and neutral sentiment categories. We found mean sentiment polarity to be approximately 0 for this no-keywords subset, with a standard deviation of around 0.39. Furthermore, dispersion within texts not containing mentions of IARM heritage is relatively low (Gini coefficient value of 0.21).

Most of the posts, comments and replies without keywords are neutral in polarity. In addition, the similar number of negative and positive texts indicates a relatively even polarity distribution across time (Figs 1–3). However, the percentage of neutral sentiment, compared to mild positive or negative sentiment, was higher from July 2013 to December 2014.

**Fig 1:** Proportion of negative, positive, and neutral texts with no IARM heritage keywords, calculated using VADER.

**Fig 2:** VADER polarity scores for the subset of the data without IARM heritage keywords. Polarity scores range from negative to positive and five categories are identified: extreme negative (<-0.75), negative (= />-0.75 and <0), neutral (0), positive (>0 and = /<0.75), and extreme positive (>0.75).

**Fig 3:** Changes in VADER polarity scores measured in six-month intervals. Percentages reflect the proportion of extreme negative, negative, neutral, positive and extreme positive scores within each six-month period. Results are shown for the subset of the data without IARM heritage keywords.

### 3.3. Follow-up investigation

Given the output of the precision-recall tests (Table 1), we relied on manual coding of Samples 1 and 2 to assess both sentiment polarity (positive or negative) and strength (mild or extreme), comparatively, for the subsets with and without references to the IARM past (Table 2). We observed that sentiment is mostly extreme, especially for the keywords subset (91% compared to 71% for no-keywords). Confirming VADER results, we find that sentiment polarity is relatively evenly split in texts without IARM heritage mentions (58% negative and 42% positive). However, sentiment polarity is mostly negative (84%) in the subset with keywords relating to the IARM past. Additionally, whereas the percentage of texts with extreme negative sentiment was only 49% in Sample 1, we find that extreme negative polarity was 92% in Sample 2.

**Table 2:** Manual coding of sentiment polarity and extremity undertaken for the precision-recall test on sampled documents from the dataset without keywords (Sample 1) and from the dataset with keywords relating to the IARM past (Sample 2).

	Extreme positive	Extreme negative	Mild positive	Mild negative
Sample 1 (N = 500)	110	245	98	47
Sample 2 (N = 300)	35	239	12	14

## 4. Discussion

After testing different methods, we identified VADER as the most accurate technique for detecting sentiment polarity and, to a lesser extent, sentiment extremity in texts that are not heritage-specific. However, none of the methods accurately captured the polarity and extremity of sentiment in politically-themed discourse on social media that includes references to the Iron Age, Roman and early medieval past. Dictionary-based methods inadequately assessed domain-specific meanings, while machine learning techniques fell short due to the unavailability of a training set of sufficient size. There are only few corpora of texts that mention ancient periods when expressing political opinions in multi-sided discussions. Integrating multiple datasets from existing and new studies of political uses of the past online may provide a way forward for future research in this area.

Generative transform and specifically large language models (LLMs) could be one way to enhance the analysis and look at more language nuances. Some studies do suggest certain limitations on richer sentiment understanding using existing LLMs, including in areas such as sarcasm [46]. Nevertheless, this is likely a promising avenue of further research as LLMs show continued improvement. Despite current shortcomings in the ability to automatically capture sentiment polarity and extremity, our manual coding strongly suggests that IARM heritage is leveraged primarily within political social media discourse characterised by negative and extreme sentiment. This result is particularly important if one considers that both VADER scores and our manual analysis found the number of positively and negatively polarised posts, comments and replies to be somewhat evenly distributed in texts without keywords related to the ancient past. The subset with heritage keywords displays an overrepresentation of negative posts, which are likely to express anger, hostility and criticism.

This finding is crucial since, as previous research has shown, the past is often invoked to express political identities [3–11]. Because such references appear in online discourse that tends to be overtly negative and heightened, they are likely to lead to motivated reasoning and polarisation [21]. Our study demonstrates that research on political identities based on social media data allows the assessment of people’s historical consciousness. However, this research over-represents individuals who relate to their present realities with negative dispositions and extreme sentiments. These conclusions should be taken into account when designing future research on heritage and identity politics.

At the same time, the differences highlighted between texts with and without IARM heritage keywords might be less prominent in analyses of different kinds of public Facebook pages or on other social media platforms. In our study, VADER results demonstrated that texts that did not contain references to the ancient past were mostly neutral. This finding is in line with the tendency towards neutral valency (average 0.56) revealed in a study of 771,036 Facebook comments from the political campaign pages Stronger In, Vote Leave, and LeaveEU for the period between 14 April 2014 and 23 June 2016 [47]. However, research by Del Vicario and colleagues [19], registered a predominantly negative sentiment for posts, comments and replies about Brexit published on the Facebook pages of news outlets. Although the discrepancy could perhaps be attributed to the different techniques deployed, it may also suggest that negative sentiment about a topic is expressed more frequently on the Facebook pages of news media outlets than on themed pages dedicated to public debates.

Furthermore, the VADER analysis we completed shows a generally even split between positive and negative sentiment in texts that did not contain keywords. These results do not align with broadly comparable analysis undertaken for Twitter. Calisir and Brambilla used the AFINN lexicon-based sentiment analyser on a corpus of tweets in English that contained the Brexit keyword and were posted between January 2016 and September 2019 [48]. They found that the number of tweets with negative sentiment was consistently higher (an average of 13 percent points) than those with positive sentiment over the period considered [48]. These findings suggest that higher proportions of negative sentiment about a particular political event are expressed on Twitter than on Facebook. To confirm this hypothesis, testing must be performed using the same sentiment analysis method to compare datasets focusing on a broader range of political issues.

## 5. Conclusion

This study demonstrates that posts that reference the ancient past in political discourse on social media are significantly more negative and more extremely polarised than those that do not contain these references. We therefore conclude that heritage keywords in politically-themed debates on social media are likely to signal the presence of more polarised and, potentially, extremist views. Furthermore, we show that social media research on political uses of the past is likely to over-represent people with very strong opinions compared to individuals whose views are more moderate.
